# Effect of Nursing Model Based on Rosenthal Effect on Self-Efficacy and Cognition of Life Meaning in Patients with Non-Small-Cell Lung Cancer

**DOI:** 10.1155/2022/6730024

**Published:** 2022-08-08

**Authors:** Linghua Mao, Huaqin Lu, Yangyang Lu

**Affiliations:** ^1^Department of Oncology, First People's Hospital of Linping District, Hangzhou, Zhejiang 311100, China; ^2^Intensive Care Unit, First People's Hospital of Linping District, Hangzhou, Zhejiang 311100, China

## Abstract

**Objective:**

To study the influence of nursing model based on Rosenthal effect on self-efficacy and cognition of life meaning in patients with non-small-cell lung cancer (NSCLC).

**Methods:**

120 patients with NSCLC treated in the hospital were selected from November 2020 to November 2021 and were randomly divided into the nursing group and the Rosenthal group, with 60 cases in each group. The nursing group received routine nursing intervention, while the Rosenthal group was intervened by nursing model based on the Rosenthal effect, and both groups were intervened for 1 month. The self-efficacy (General Self-Efficacy Scale (GSES)), negative emotions (Hospital Anxiety and Depression Scale (HADS)), self-burden (Self-Perceived Burden Scale for Cancer Patients (SPBS-CP)), meaning of life (Meaning of Life Scale for Advanced Cancer Patients (MiLS)), and quality of life (Functional Assessment of Cancer Therapy-Lung (FACT-L)) were compared between the two groups before and after intervention.

**Results:**

After 1 month of intervention, the scores of GSES and MiLS of patients in the two groups were significantly higher than those before intervention, and the scores in the Rosenthal group were significantly higher than those in the nursing group (*P* < 0.05). The scores of HADS, SPBS-CP, and FACT-L in the two groups were significantly lower than those before intervention, and the scores were significantly lower in the Rosenthal group than those in the nursing group (*P* < 0.05).

**Conclusion:**

Nursing model intervention based on Rosenthal effect enhances the self-efficacy and meaning of life and reduces the negative emotions and self-burden in patients with NSCLC.

## 1. Introduction

Lung cancer is one of the three major tumor diseases in the world, and about 80% of lung cancer patients have non-small-cell lung cancer (NSCLC). The incidence of NSCLC is related to poor air quality, living and working environment, etc., of which the incidence is increasing year by year [1]. Radiotherapy and chemotherapy are the conventional treatment approaches of NSCLC; however, the treatment courses of radiotherapy and chemotherapy are long with high toxicity, side effects, and high cost. All the above disadvantages will bring psychological pressure and self-burden to patients, inducing negative emotions in patients and even having a negative impact on treatment and suicide. Therefore, appropriate psychological intervention is needed to alleviate the negative emotions [2, 3]. Psychotherapy is a green medicine for cancer rehabilitation, and there is no toxic side effect, but it has the irreplaceable function of surgery, chemotherapy, and radiotherapy; a person's heart is full of anxiety and fear of death, despair of survival, and internal ecosystem disorders will occur obviously. The effect will be half the effort. Routine nursing interventions help patients release negative emotions through psychological counseling; however, the outcome is poor, as the patients lose their life expectancy and the meaning of life [4]. The Rosenthal effect enables patients to gain positive emotions through psychological cues such as praise, encouragement, and trust, which is mostly used in patients with advanced cancer [5]. This study uses a care model based on the Rosenthal effect to intervene in the treatment of NSCLC patients and observe the effect.

## 2. Materials and Methods

### 2.1. General Data

A total of 120 NSCLC patients admitted to our hospital from November 2020 to November 2021 were selected and randomly divided into the nursing group and the Rosenthal group with 60 cases in each group. Inclusion criteria were as follows: diagnosed with NSCLC [6]; expected survival >1 month; and normal communication. Exclusion criteria were as follows: severe mental illness; combined with primary malignant tumors in other parts; and combined with liver, kidney, heart, and other important organ dysfunction and other diseases. There was no significant difference in the general data of the two groups of patients (*P* < 0.05) (Table 1).

## 3. Method

Routine nursing interventions were used in patients of the nursing group, including NSCLC-related health education, psychological counseling, and so on. Nursing staff communicated with NSCLC patients and their families to understand their emotional and psychological states, helped patients release negative emotions by using patient listening and other methods, and tried to meet the needs of NSCLC patients as conditions permit.

A nursing model intervention based on the Rosenthal effect was used in the Rosenthal group. (1) Before the treatment, when the patient is admitted to the hospital, the nursing staff will register his personality, preferences, illness, treatment situation, etc. and establish a personal health file. Nursing staff introduced the relevant knowledge of NSCLC pathogenesis to patients and their relatives in detail and emphasized the importance of positive attitude for treatment and nursing. During the explanation, the educational level of patients is considered by the nurses to facilitate the patient's understanding and acceptance of the explanation method. Examples are used to explain the correlation between psychological state, treatment effect, and disease outcome. Patients were instructed to express their feelings to nurses or family members in a timely manner. (2) After the treatment starts, ① nursing staff randomly divide NSCLC patients into groups, with about 10 patients as a group, and give lectures as well as communication activities regularly. Nursing staff explain the importance of physical and mental health during lectures, encourage patients to tell their own stories about illness, treatment, psychological thoughts, etc., and encourage patients to conduct self-evaluation. Encourage patients to evaluate themselves positively and instruct group patients to positively encourage and praise others. In group activities, nurses try to invite family members of NSCLC patients to participate in live or participate in short video, voice, etc., guide patients to review positive things in the treatment process or things that they are encouraged and supported, and gradually guide patients to expand their positive impact and significance. Nursing staff invite patients with positive attitudes to give speeches, share their feelings, skills, and experiences in maintaining their positive emotions and mentality. Organize patients to discuss, exchange, and share their own experiences with each other. ② Continuously observe the toxic and side effects of patients with NSCLC and inform the patients and their families of coping methods. Communicate with patients weekly to understand changes in their state of mind and use “Are you confident to persist in treatment and why”? Putting forward some questions, such as “which” to guide the patient to review and think, patiently listen to the patient's expression, and appropriately use affirmation particles and body movements to support the patient. Encourage patients to express positive psychological emotions and thoughts during the treatment process and guide patients to self-affirmation, such as “I can definitely achieve a certain goal,” “I can definitely adhere to the treatment,” and so on. ③ Establish an online communication platform, such as WeChat group, invite the attending doctor, nursing staff, NSCLC patients, and their family members to participate and share the relevant knowledge of NSCLC and treatment of toxic and side effects in the group regularly, as well as how to self-discharge negative emotions, and set up psychological counseling personnel to give patients psychological counseling at any time. Both groups were treated for 1 month.

### 3.1. Observation Indicators

(1) Self-efficacy: the General Self-Efficacy Scale (GSES) [7] was used to evaluate and compare the self-efficacy of the two groups of patients before and after the intervention, including 10 items, each of which was scored 1–4 points, respectively, with a full score of 40. The higher the score, the higher the patient's self-efficacy. (2) Negative emotions: the Hospital Anxiety and Depression Scale (HADS) [8] was used to evaluate and compare the negative emotions of the two groups of patients before and after the intervention. Seven categories of anxiety and depression were included, each with a score of 0–3, and the higher the score is, the more negative emotions the patient had. (3) Self-burden: the self-burden evaluation scale of Chinese cancer patients (SPBS-CP) [9] was used to evaluate and compare the self-burden of the two groups of patients before and after the intervention, including a total of 21 items in 4 aspects of care, economy, psychology, and treatment. 5-level scoring is used for each item. Scores <30 indicate no obvious burden, 30≤score <50 indicates mild burden, 50≤score <70 indicates moderate burden, and score ≥70 indicates severe burden. High indicates that the patient feels more self-burdened. (4) Sense of meaning in life: the Meaning Of Life Scale (MiLS) [10] in patients with advanced cancer was used to evaluate and compare the sense of meaning in life of the two groups of patients before and after the intervention, including 4 items of will, 5 items of frustration, 4 items of satisfaction, and 7 items of control. There are 4 items of tolerance, 4 items of acceptance and 6 dimensions, and each item is scored on a 5-point scale. Higher score indicates stronger sense of life meaning of the patients. (5) Quality of life: the quality of life of patients with lung cancer (FACT-L) [11] was used to evaluate and compare the quality of life of the two groups of patients before and after the intervention, including 7 items of physiology, 7 items of function, 6 items of emotion, and 9 items of additional attention, each using a 5-level score; the lower the score, the higher the quality of life of the patient.

### 3.2. Statistical Methods

SPSS 22.0 was used for statistics, count data were expressed as %, *χ*2 test was performed, rank-sum test was performed between rank data groups, measurement data were expressed as ± *s*, and *t*-test was performed. *P* < 0.05 was considered statistically significant.

## 4. Results

### 4.1. Comparison of Self-Efficacy and Negative Emotions between the Two Groups after 1 Month of Intervention

The GSES scores of the two groups of patients were significantly higher than those before the intervention, and the scores of the Rosenthal group were significantly higher than those of the nursing group (*P* < 0.05); The HADS scores of the patients in the two groups were significantly lower than those before the intervention, and the scores of the patients in the Rosenthal group were significantly lower than those in the nursing group (*P* < 0.05), as shown in Table 2.

### 4.2. Comparison of Self-Burden Sense between the Two Groups of Patients

After 1 month of intervention, the SPBS-CP scores in the two groups were significantly lower than those before the intervention, and the scores in the Rosenthal group were significantly lower than those in the nursing group (*P* < 0.05), as shown in Table 3.

### 4.3. Comparison of the Meaning of Life between the Two Groups of Patients

After 1 month of intervention, the MiLS scores in the two groups were significantly higher than those before the intervention, and the scores in the Rosenthal group were significantly higher than those in the nursing group (*P* < 0.05), as shown in Table 4.

### 4.4. Comparison of Quality of Life between the Two Groups of Patients

After 1 month of intervention, the FACT-L scores of the patients in the group were significantly lower than those before the intervention, and the scores of the patients in the Rosenthal group were significantly lower than those in the nursing group (*P* < 0.05), as shown in Table 5.

## 5. Discussion

With the development of medical technology, the 5-year survival rate of NSCLC patients has gradually increased. However, during the process of treatment, diseases, side effects of treatment, and economic pressure will cause psychological pressure to patients and increase their sense of self-burden, which induces patients to consider treatment care and life negatively and affects the outcomes of treatment and care. It is critical to use scientific and appropriate interventions to improve the psychological state of patients [12].

In our study, NSCLC was classified using TNM staging. This staging may be associated with pretreatment clinical staging, pathological staging, postoperative staging, post-neoadjuvant staging, or post-neoadjuvant and surgical staging. Clinical staging before treatment is based on a combination of history, clinical examination, serology, diagnostic imaging, endoscopic evaluation, diagnostic surgical evaluation, and pathology. Accurate staging and scoring of the fitness status of patients with NSCLC are critical for prognosis and treatment planning.

The toxic and side effects, disease, and economic pressure caused by NSCLC patients receiving radiotherapy and chemotherapy for a long time increase their sense of self-burden, causing many patients to have excessive anxiety, depression, and other negative emotions, resulting in a decrease in their sense of self-efficacy and meaning of life, which in turn affects the treatment progress and effects [13]. Although routine nursing interventions provide psychological counseling to patients and help patients release negative emotions, it is difficult to correct patients' negative thoughts and psychological states, resulting in a strong sense of self-burden and a low sense of self-efficacy and meaning in life [14]. The Rosenthal effect is to use positive evaluation methods such as praise and encouragement to help patients restore self-confidence and self-esteem [15]. In the results of this study, after 1 month of intervention, the GSES and MiLS scores of the two groups of patients were significantly higher than those before the intervention, and the scores of the Rosenthal group were significantly higher than those of the nursing group, and the HADS and SPBS-CP scores of the two groups were obviously lower than those of the nursing group. Before intervention, the scores of patients in the Rosenthal group were significantly lower than those in the nursing group, suggesting that the nursing model based on the Rosenthal effect intervening in NSCLC patients can effectively relieve their negative emotions, reduce their sense of self-burden, and enhance self-efficacy, life expectancy, and sense of meaning of patients. The reason is that in the nursing model based on the Rosenthal effect, before the start of the patient's treatment, the nurses fully understand the personality of patients, preferences, and other basic information, conduct health education in a way that the patient is easy to accept, and help the patient understand the relationship between the psychological state and the treatment effect. They provide health education in a way that is easy for patients to understand, help patients understand the correlation between psychological status and treatment outcomes, and prepare patients for subsequent psychological adjustments [16]. After the treatment begins, the nurses divide the patients into a group mode, organize the NSCLC patients between the groups to share their disease and treatment feelings, and guide the patients themselves, their families, and members of the group to make positive evaluations, so as to help the patients gain a sense of emotional belonging and support. It can effectively enhance self-efficacy of patients and reduce their self-burden [17]. Nursing staff establish a good emotional outlet for NSCLC patients in the mode of group communication, help patients vent their negative emotions through expressions, and guide other patients to encourage other patients in a timely manner, so as to effectively relieve the anxiety and depression of NSCLC patients. Nursing staff invite patients with good and positive attitude to give speeches to stimulate the emotions and attitudes of other patients, encourage, and support each other, thereby effectively improving their sense of meaning in life [18].

Negative emotions and physical and mental stress of NSCLC patients will affect their treatment effect and even increase the toxic and side effects of radiotherapy and chemotherapy, affect their physical and mental status, increase the burden on patients' families, and reduce their quality of life [19]. Routine nursing intervention is difficult to correct the negative emotions of patients, resulting in insufficient self-efficacy and meaning of life and negative treatment of survival and treatment, affecting their quality of life. In the results of this study, the FACT-L score of the patients in the 1-month intervention group was significantly lower than that before the intervention, and the scores of the patients in the Rosenthal group were significantly lower than those in the nursing group, indicating that the nursing model based on the Rosenthal effect intervenes in patients with NSCLC and can improve the quality of life of patients. Because basing on the Rosenthal nursing model, the encourages, praises, and supports from other NSCLC patients, their family members, and nurses, which can enable NSCLC patients to fully feel the care of others and organize patients to exchange experiences and ideas with each other. Also, it can help them to improve their sense of self-efficacy, reduce their sense of self-burden, improve their psychological state, which is beneficial for patients to actively face treatment and nursing, provide guarantee for treatment and nursing effects, relieve physical discomfort caused by diseases and toxic side effects, and eventually improve life quality of patients [20].

In conclusion, intervening patients with NSCLC through a nursing model based on the Rosenthal effect reduces the negative emotions and burden, improves self-efficacy and meaning sense of life, and improves quality of life of the patients, which is valuable for clinical application.

## Figures and Tables

**Table 1:** General data.

Indexes	Number of cases	
Gender	Nursing group	Rosenthal group
Male	31	32
Female	29	28
Age	22–67 (44.72 ± 10.85) years	23–66 (44.10 ± 10.67) years
The course of disease	6 months–2 years	5 months–2 years
TNM staging		
Stage II	20	22
Stage III	23	24
Stage IV	17	14
Types of NSCLC		
Squamous-cell carcinoma	21	22
Adenocarcinoma	16	17
Large-cell carcinoma	23	21

**Table 2:** Comparison of self-efficacy and negative emotions in the two groups before and after intervention (*n* = 60, points, ±*s*).

Group	Time	GSES	HADS	
			Anxiety	Depressed
Rosenthal group	Before intervention	21.88 ± 4.35	16.52 ± 3.39	16.11 ± 3.25
	After intervention	32.15 ± 3.21^a^	7.49 ± 2.23^a^	7.39 ± 2.36^a^
Nursing group	Before intervention	22.06 ± 4.49	16.83 ± 3.42	15.90 ± 3.31
	After intervention	30.47 ± 3.06^a^	8.92 ± 2.61^a^	8.80 ± 2.78^a^
*t *_after intervention_		2.934	3.227	2.995
*P *_after intervention_		0.004	0.002	0.003

*Note.* Compared with before intervention, ^a^*P* < 0.05。.

**Table 3:** Comparison of self-burden before and after intervention in the two groups (*n* = 60, cases, %).

Group	Time	No obvious burden	Mild burden	Moderate burden	Severe burden
Rosenthal group	Before intervention	0 (0.00)	8 (13.33)	25 (41.67)	27 (45.00)
	After intervention	8(13.33)^a^	35 (58.33)^a^	10 (16.67)a	7 (11.67)^a^
Nursing group	Before intervention	0(0.00)	7 (11.67)	24 (40.00)	29 (48.33)
	After intervention	4 (6.67)^a^	26 (43.33)^a^	17 (28.33)^a^	13 (21.67)^a^
*Z* after intervention	2.440				
*P* after intervention	0.015				

*Note.* Compared with before intervention, ^a^*P* < 0.05.

**Table 4:** Comparison of the meaning of life in the two groups before and after the intervention (*n* = 60, points, ±*s*).

Group	Time	Will	Frustration	Satisfy	Control	Bear	Accept
Rosenthal group	Before intervention	6.28 ± 1.33	7.91 ± 1.78	6.25 ± 1.31	13.97 ± 2.52	6.52 ± 1.42	6.48 ± 1.37
	After intervention	13.84 ± 2.46^a^	17.99 ± 3.56^a^	13.79 ± 2.31^a^	26.81 ± 4.39^a^	13.55 ± 2.29^a^	13.67 ± 2.40^a^
Nursing group	Before intervention	6.09 ± 1.26	7.64 ± 1.70	6.38 ± 1.34	14.35 ± 2.61	6.64 ± 1.49	6.67 ± 1.42
	After intervention	12.47 ± 2.19^a^	16.51 ± 3.16^a^	12.65 ± 2.12^a^	24.72 ± 4.05^a^	12.53 ± 2.01^a^	12.66 ± 2.19^a^
	*t *_after intervention_	3.222	2.408	2.816	2.710	2.593	2.408
	*P *_after intervention_	0.002	0.018	0.006	0.008	0.011	0.018

*Note.* Compared with before intervention, ^a^*P* < 0.05.

**Table 5:** Comparison of the quality of life between the two groups before and after intervention (*n* = 60, points, ±*s*).

Group	Time	Physiological	Features	Emotion	Additional attention
Rosenthal group	Before intervention	20.16 ± 3.35	19.88 ± 3.26	16.49 ± 2.79	26.78 ± 4.31
	After intervention	11.43 ± 2.51^a^	10.79 ± 2.44^a^	8.83 ± 2.11^a^	14.99 ± 2.95^a^
Nursing group	Before intervention	20.84 ± 3.41	19.12 ± 3.34	16.85 ± 2.83	27.57 ± 4.50
	After intervention	12.58 ± 2.69^a^	12.26 ± 2.61^a^	9.70 ± 2.34^a^	16.63 ± 3.26^a^
	*t *_after intervention_	2.421	3.187	2.139	2.889
	*P *_after intervention_	0.017	0.002	0.035	0.005

*Note.* Compared with before intervention, ^a^*P* < 0.05.

## Data Availability

The data used to support the findings of this study are available from the corresponding author upon request.
